# Analysis of the Dose Drop at the Edge of the Target Area in Heavy Ion Radiotherapy

**DOI:** 10.1155/2021/4440877

**Published:** 2021-11-11

**Authors:** Xiaoyun Ma, Mengling Zhang, Wanbin Meng, Xiaoli Lu, Ziheng Wang, Yanshan Zhang

**Affiliations:** ^1^Department of Medical Physics, Wuwei Tumor Hospital Heavy Ion Therapy Center, No. 31 Sanitary Lane, Haizang Road, Wuwei City, Gansu Province, China 733000; ^2^Department of Heavy Ion Radiotherapy, Wuwei Tumor Hospital, No. 31 Sanitary Lane, Haizang Road, Wuwei City, Gansu Province, China 733000

## Abstract

**Background:**

The dose distribution of heavy ions at the edge of the target region will have a steep decay during radiotherapy, which can better protect the surrounding organs at risk.

**Objective:**

To analyze the dose decay gradient at the back edge of the target region during heavy ion radiotherapy.

**Methods:**

Treatment planning system (TPS) was employed to analyze the dose decay at the edge of the beam under different incident modes and multiple dose segmentation conditions during fixed beam irradiation. The dose decay data of each plan was collected based on the position where the rear edge of the beam began to fall rapidly. Uniform scanning mode was selected in heavy ion TPS. Dose decay curves under different beam setup modes were drawn and compared.

**Results:**

The dose decay data analysis showed that in the case of single beam irradiation, the posterior edge of the beam was 5 mm away, and the posterior dose could drop to about 20%. While irradiation in opposite direction, the posterior edge of the beam was 5 mm away, and the dose could drop to about 50%. In orthogonal irradiation of two beams, the posterior edge of the beam could drop to about 30-38% in a distance of 5 mm. Through the data analysis in the TPS, the sharpness of the dose at the back edge of the heavy ion beam is better than that at the lateral edge, but the generated X-ray contamination cannot be ignored.

**Conclusions:**

The effect of uneven CT value on the dose decay of heavy ion beam should also be considered in clinical treatment.

## 1. Introduction

Surgery, radiotherapy, and chemotherapy are three main methods for treating cancer, among which radiotherapy plays an increasingly prominent role in tumor treatment [1]. Approximately 70% of cancer patients are subjected to radiotherapy, and some of them could be cured by radiotherapy [2, 3].

Traditional radiotherapy mainly utilizes X-rays and electron rays produced by medical electron linear accelerators or various kinds of X-ray therapy machines to irradiate part of the tumor and kill it. The efficacy of traditional radiotherapy depends on the radiosensitivity of the tumor [4]. Subsequently, it has been found that compared with other conventional rays (X-rays, *γ* rays, electron lines, proton lines, neutron lines, *π*-meson lines, etc.), charged heavy ions have unique advantages in the treatment of cancer due to their physical and biological characteristics. Heavy ions, also known as Bragg peak, are the ions with an atomic number of 2 or greater and have lost their electrons [5]. When charged heavy ions pass through human tissues, the dose curve remains relatively constant at the shallow layer, forming a low dose flat region [6]. Compared with X-rays, heavy ions have relatively high relative biological effectiveness (RBE) in the Bragg peak region, which is considered as a good radiotherapy beam to kill tumor cells in the target region and protect the normal tissues around and on the radiation path as much as possible to reduce their damage [7, 8].

Heavy ion treatment plans often require only two or three beams to meet clinical prescription requirements [9–11]. For fixed nozzle treatment, we usually use single beam irradiation, two-beam opposite irradiation, and two-beam orthogonal irradiation. Beam delivery is the process of transporting heavy ion beam from accelerator to target area for irradiation therapy. During the active beam delivery, the accelerator actively changes the energy of the particles to change the incidence depth of the ion beam [12]. Meanwhile, the magnetic scanning system is used to guide the pencil beam to carry out conformal or intensity-modulated irradiation therapy on the tumor target region. In order to reduce the number of stratified irradiations and shorten the irradiation time, the active pencil beam spot was scanned [13].

When the passive scanning beam is delivered, the accelerator provides a beam of fixed energy, which is broadened laterally into a large irradiation field by scanning the magnet and the scatterer [14]. The ridge filter lengthwise broadens the sharp peak of the single energy beam to the Bragg peak which is consistent with the thickness of the tumor. A range shifter is placed along the beam path to adjust the beam energy to reach different incident depths [15].

Uniform scanning is one of the passive beam delivery mode, when heavy ions are applied in clinical radiotherapy, which adopts triangular wave scanning mode to extend the beam laterally, ridge filter to lengthwise expand the Bragg peak of the beam, and combined with a lobed collimator to carry out lateral conformal irradiation [16]. In our literature, we analyze the beam mode, under the condition of multiple doses split on the edge of the target dose drop speed, for heavy ion radiotherapy, provide reference for clinicians treating patients with data, and can also be used for delineation, relatively safe distance between target and endanger organ to provide the reference data.

## 2. Materials and Methods

### 2.1. Data Acquisition

Data acquisition was used heavy ion treatment planning system (TPS). The version of TPS is ciPlan1.0, made by Lanzhou KJTJ New Technology Co., Ltd., China. The principle of the heavy ion TPS is the use of computed tomography (CT) as the basic input data, extracting CT value (Hounsfield unit (HU)), conducted on the CT value along the beam through the direction of water after the equivalent transformation, the use of biological models, calculation of heavy ions in the human body or medium range, energy deposition, and dose distribution. The TPS based on microcomputer Microsoft Visual C++ program to simulate the accelerating field (accelerated circulation), deflection and focusing magnetic field and other corresponding equipment features, cooperate with the ridge type filters and drop can call, and digital control beam spot size, beam nominal energy and Bragg peak stretcher, collimator built-in mortise and tenon joint structure of the multimedia tungsten copper alloy blade, consistent with the treatment of terminal compatibility. The built-in algorithm builds a model based on the dose Bragg peak distribution characteristics of HIM high-energy carbon ion (^12^C^6+^) beam in aqueous medium and uses the dose pen beam algorithm (pencil beam calculation (PBC)) principle. The TPS includes parameters of equipment, such as nozzles in the treatment room, energy range, beam radial dose distribution, and relative biological effect ratio statistics. This TPS can realize the basic functions, such as patient positioning CT import, image fusion, target and normal organs contouring, plan designing, plan comparison, treatment plan reports export, and QA mode.

### 2.2. Methods

To set a uniform water cube phantom in heavy ion TPS, the field size is 10 cm × 10 cm. Uniform scanning mode was selected in TPS, then to design multiple heavy ion treatment plans with single beam irradiation, two-beam irradiation in opposite direction, and two-beam orthogonal irradiation under common segmentation conditions. Measuring dose change data, on the end edge of the beam at the center of the beam axis, using 95% isodose line position as a benchmark, define its dosage as 100% and 0 mm distance. Then, the dose data of each point in the 20 mm distance are measured. We collected dose decay data of standard plans with 20, 15, 10, and 6 fractions with total dose of 60 Gy (RBE). The statistics are shown in Table 1.

It can be seen from Table 1 that the dose decay trend makes no difference in the same irradiation mode under different fractionation conditions. When using single beam irradiation, the heavy ion dose can quickly drop to about 50%-60% of the prescribed dose, at the position of 3 mm away from the 95% isodose line, in the trailing edge of the center axis. The dose can drop to about 20%-30% 5 mm away. X-ray of traditional radiotherapy can never decay so steeply in 5 mm. This significant characteristic enables heavy ion therapy for difficult cases where the organs at risk are close to the target region. When designing the treatment plan, the medical physicist can reduce the dose of the adjacent organs to the constrain on the basis of reaching the target prescription dose.

## 3. Results

1. *Dose Decay Curve under Different Beam Setup Modes*. To select the plans of 4 Gy (RBE) per fraction in the TPS to compare the dose decay curves of different beam setup modes, as shown in Figure 1

As shown in Figure 1, the dose decay is most steeply in single beam exposure, which shows the characteristic of dose decay of the heavy ion directly. Dose dropped slowest during two beams; this is due to multiple Bragg peaks' plateau dose overlay in heavy ion SOBP, resulting a relative high dose in the front edge of the SOBP. Meanwhile, when using two beams, the dose in a relatively far distance also maintains a high level (20 mm position was greater than 35%) that is the same reason. The trailing edge of one orthogonal field is the side edge of the other field, and the dose is the superposition of the penumbra of the trailing edge of Bragg peak and the dose edge. Compared with the trailing edge of simple Bragg peak, the drop rate is slightly slower, and the distance to the gentle area is longer. Beam dose curve flattens out after steep fall in the flat area. The dose of trailing edge of two-beam orthogonal irradiation is lower than single beam, it is because that the heavy ion beam can produce X-ray contamination behind the Bragg peak during passing through the tissue [17]. The Bragg peak forms a “tail”, because of the contribution of the X-ray contamination. Due to the lateral scattering X-ray quantity is less, the beam lateral edge does not exist in this such low dose area. The double beams orthogonal irradiation superimposes the dose of the trailing edge and the lateral edge of the beam. In the case of two-beam weight 1 : 1, the dose in the low-dose area behind the single beam is almost twice that behind the double-beam orthogonal radiation.

(2) *Dose Decay Curves in Different Fractions*. For each beam setup irradiation mode, draw a comparison chart of dose decay curve in different fractions, respectively, shown in Figures 2–4

It can be seen that under the same irradiation mode, the dose decay curve trend of different fractions is basically the same. The overall dose was slightly higher in the hypofractionation (10 Gy (RBE)) for a single fraction, especially in the single beam irradiation and two-beam irradiation in opposite direction, which may because of the greater X-ray contamination caused by the higher dose, which still needs to be confirmed by actual measurement.

## 4. Discussion

When a heavy ion beam is used for radiotherapy, because of its unique physical characteristics, the dose at the edge of the target area falls very rapidly as revealed in the analysis of the data in the planning system. The trailing edge of the heavy ion beam center is removed from the 95% isodose line by 5 mm, at which the dose can be reduced to approximately 20-30% of the prescription dose; that is, at 5 mm, the dose can be reduced by 70-80%, which is the key advantage of heavy ion therapy. This makes it possible for heavy ions to safely treat patients with tumors close to endangered organs.

One study compared the drop in dose gradient at the edge of the target area for five kinds of equipment (wave knife, spiral tomography therapy (Tomo), edge accelerator, trilogy accelerator, and gamma knife) in stereotactic radiotherapy for pancreatic cancer when using X/*γ* rays for radiotherapy. The authors concluded that all five kinds of radiotherapy equipment are capable of completing the stereotactic radiotherapy plan for pancreatic cancer that meets the clinical requirements. Among them, the wave knife and gamma knife had better dose drop gradients [18]. In another study, stereotactic radiotherapy (SBRT) was used to treat vertebral metastases using a radiosurgery system. The relative dose drop rate in the spinal cord direction was analyzed. The authors concluded that the relative dose drop in the 40 Gy group was 0.87 ± 0.60 mm/5% Dmax and that in the 33 Gy group was 0.69 ± 0.16 mm/5% Dmax. From these studies, it can be seen that the dose drop rate for stereotactic radiotherapy is faster when using X/*γ* ray radiotherapy, and the radiation knife and gamma knife have better dose drop gradients of approximately 5% at 0.8 mm. However, the dose of the heavy ion beam can be reduced by approximately 8%-19% 1 mm away from the 95% isodose line, at the trailing edge of the field. Consequently, the dose drop rate of the heavy ion beam remains the fastest. This allows the heavy ion beam to treat difficult cases where the endangered organ is very close to the target area. The physicist can reduce the dose to the adjacent endangered organ to within the limit while meeting the dose requirements of the target area when designing the treatment plan.

In practice, human tissue is not uniformly irradiated by the heavy ion beam; the data analyzed in this paper were obtained from the heavy ion treatment planning system using a treatment plan designed in a uniform water phantom. The calculation of measurements in the planning system is based on CT values, and the uneven tissue in the human body will also affect the dose drop curve behind the field in the actual treatment of heavy ion patients. It is also necessary to use the actual calculated values in the planning system as a reference and fully consider the positional relationship with the adjacent endangered organs when drawing the target area. As a result, when the target area reaches the prescription dose, the radiation dose of the adjacent endangered organs is also ensured to be within the clinically acceptable range [19].

A heavy ion radiotherapy system is expensive. Consequently, heavy ion radiotherapy is often used to treat more recurrent tumors after conventional radiation therapy and for patients who are unable to undergo conventional radiotherapy because the tumor is especially close to endangered organs. The effective and safe treatment of these patients is a challenge to heavy ion doctors and physicists. There are few reports on the dose drop rate at the edge of the target area during heavy ion radiotherapy at present. The results can provide reference data for the clinical application of heavy ion beams.

## Figures and Tables

**Figure 1:** Comparison of dose decay curves under different beam setup modes. The plans of 4 Gy (RBE) per fraction in the TPS were selected to compare the dose decay curves of different beam setup modes. Multiple heavy ion treatment plans with single beam irradiation, two-beam irradiation in opposite direction, and two-beam orthogonal irradiation under common segmentation conditions were designed in a homogeneous water phantom.

**Figure 2:** Dose decay curves in different fractionations (single beam irradiation). Multiple heavy ion treatment plans with single beam irradiation, two-beam irradiation in opposite direction, and two-beam orthogonal irradiation under common segmentation conditions were designed in a homogeneous water phantom.

**Figure 3:** Dose decay curves in different fractionations (two-beam irradiation in opposite direction). Multiple heavy ion treatment plans with two-beam irradiation in opposite direction under common segmentation conditions were designed in a homogeneous water phantom.

**Figure 4:** Dose decay curves in different fractionations (two-beam orthogonal irradiation). Multiple heavy ion treatment plans with two-beam orthogonal irradiation under common segmentation conditions were designed in a homogeneous water phantom.

**Table 1:** Dose decay data at the end edge of beam.

Parameters of TPS			Dose decay percentage at the end edge of beam (at a specified distance: mm)							
Beam setup	Fractions	Dose/Fx Gy (RBE)	1 mm	2 mm	3 mm	4 mm	5 mm	10 mm	15 mm	20 mm
Single direction beam	20	3	86.43%	66.10%	45.78%	25.46%	18.84%	16.95%	15.51%	14.13%
	15	4	81.81%	61.87%	41.93%	24.20%	19.95%	17.98%	16.49%	15.03%
	10	6	91.60%	72.17%	52.73%	33.29%	22.52%	20.20%	18.52%	16.94%
	6	10	84.22%	65.69%	47.16%	29.81%	25.43%	23.07%	21.24%	19.45%

Two-beam irradiation in opposite direction	20	3	92.13%	78.75%	65.37%	51.99%	45.93%	41.30%	38.00%	35.41%
	15	4	91.66%	78.57%	65.47%	52.38%	47.02%	42.40%	39.10%	36.49%
	10	6	93.27%	80.69%	68.11%	55.53%	49.14%	44.52%	41.18%	38.52%
	6	10	88.25%	76.49%	64.74%	54.45%	52.07%	47.60%	44.31%	41.65%

Horizontal and vertical (horizontal beam)	20	3	90.88%	76.16%	61.43%	46.91%	36.62%	9.93%	7.34%	6.68%
	15	4	91.36%	76.79%	62.22%	47.66%	37.40%	10.27%	7.63%	6.94%
	10	6	91.18%	76.92%	62.65%	48.58%	38.29%	10.83%	8.13%	7.41%
	6	10	86.01%	72.03%	58.04%	45.04%	36.75%	11.45%	9.03%	8.24%

Horizontal and vertical (vertical beam)	20	3	86.30%	70.17%	54.04%	37.96%	30.34%	10.16%	7.54%	6.88%
	15	4	83.90%	67.80%	51.70%	35.76%	29.88%	10.34%	7.83%	7.16%
	10	6	85.38%	69.57%	53.77%	38.71%	31.18%	10.96%	8.31%	7.60%
	6	10	84.35%	68.70%	53.06%	38.22%	32.06%	11.88%	9.24%	7.62%

## Data Availability

The data used during the present study are available from the corresponding author upon reasonable request.
